The article "Hypertonic Saline Compared to Mannitol for the Management of Elevated Intracranial Pressure in Traumatic Brain Injury: A Meta-Analysis" was retracted in 2023. Reasons: plagiarism; overlap with other authors' work; unreliable results or conclusions; concerns about the authorship.

# Hypertonic Saline Compared to Mannitol for the Management of Elevated Intracranial Pressure in Traumatic Brain Injury: A Meta-Analysis

**DOI:** 10.3389/fsurg.2021.765784

**Published:** 2022-01-07

**Authors:** Chengchen Han, Fan Yang, Shengli Guo, Jianning Zhang

**Affiliations:** ^1^Department of Neurosurgery, The Sixth Medical Center of PLA General Hospital, Beijing, China; ^2^Department of Neurosurgery, The First Medical Center of PLA General Hospital, Beijing, China

**Keywords:** hypertonic saline, mannitol, intracranial pressure, treatment failure, cerebral perfusion pressure, traumatic brain injury, favorable outcome, mortality

## Abstract

**Background:** We performed a meta-analysis to evaluate the effect of hypertonic saline compared to mannitol for the management of elevated intracranial pressure in traumatic brain injury.

**Methods:** A systematic literature search up to July 2021 was performed and 17 studies included 1,392 subjects with traumatic brain injury at the start of the study; 708 of them were administered hypertonic saline and 684 were given mannitol. They were reporting relationships between the effects of hypertonic saline compared to mannitol for the management of elevated intracranial pressure in traumatic brain injury. We calculated the odds ratio (OR) and mean difference (MD) with 95% confidence intervals (CIs) to assess the effect of hypertonic saline compared to mannitol for the management of elevated intracranial pressure in traumatic brain injury using the dichotomous or continuous method with a random or fixed-effect model.

**Results:** Hypertonic saline had significantly lower treatment failure (OR, 0.38; 95% CI, 0.15–0.98, *p* = 0.04), lower intracranial pressure 30–60 mins after infusion termination (MD, −1.12; 95% CI, −2.11 to −0.12, *p* = 0.03), and higher cerebral perfusion pressure 30–60 mins after infusion termination (MD, 5.25; 95% CI, 3.59–6.91, *p* < 0.001) compared to mannitol in subjects with traumatic brain injury.

However, hypertonic saline had no significant effect on favorable outcome (OR, 1.61; 95% CI, 1.01–2.58, *p* = 0.05), mortality (OR, 0.59; 95% CI, 0.34–1.02, *p* = 0.06), intracranial pressure 90–120 mins after infusion termination (MD, −0.90; 95% CI, −3.21–1.41, *p* = 0.45), cerebral perfusion pressure 90–120 mins after infusion termination (MD, 4.28; 95% CI, −0.16–8.72, *p* = 0.06), and duration of elevated intracranial pressure per day (MD, 2.20; 95% CI, −5.44–1.05, *p* = 0.18) compared to mannitol in subjects with traumatic brain injury.

**Conclusions:** Hypertonic saline had significantly lower treatment failure, lower intracranial pressure 30–60 mins after infusion termination, and higher cerebral perfusion pressure 30–60 mins after infusion termination compared to mannitol in subjects with traumatic brain injury. However, hypertonic saline had no significant effect on the favorable outcome, mortality, intracranial pressure 90–120 mins after infusion termination, cerebral perfusion pressure 90–120 mins after infusion termination, and duration of elevated intracranial pressure per day compared to mannitol in subjects with traumatic brain injury. Further studies are required to validate these findings.

The article "Hypertonic Saline Compared to Mannitol for the Management of Elevated Intracranial Pressure in Traumatic Brain Injury: A Meta-Analysis" was retracted in 2023. Reasons: plagiarism; overlap with other authors' work; unreliable results or conclusions; concerns about the authorship.

## Introduction

Traumatic brain injury is one of the main reasons for death and disability in the world. Generally, the frequency of traumatic brain injury in Europe is >2,000 per million yearly (1). Increased intracranial pressure is very common after severe traumatic brain injury and is frequently triggered by brain edema (2). As high intracranial pressure is related to increased death and impaired functional results (3), controlling intracranial pressure is a major constituent of traumatic brain injury treatment (2). Guidelines suggest more conservative interventions, e.g., raise of the upper body, cerebrospinal fluid drainage, and the use of hypnotics and hyperosmolar solutions before executing decompressive craniectomy (4–6). Osmotic agents are used to reducing elevated intracranial pressure, improve cerebral perfusion pressure, and presumably improve cerebral blood flow. Yet, osmotic agents have other physiological effects that can influence cerebral blood flow (7). There are a lot of studies that confirmed its use in the management of intracranial pressure after traumatic brain injury (8–11). hypertonic saline and mannitol are examples of those osmotic agents used in the management of intracranial pressure after traumatic brain injury (12–14). The intracranial pressure-decreasing properties of mannitol and hypertonic saline are well known (15), but the clinical advantage of one over the other has not been confirmed. However, mannitol is being often used for the management of high intracranial pressure; up-to-date drug-approval procedures have never been shown. Though animal trials recommend benefits of hypertonic saline over mannitol e.g., reduced neuroinflammatory activity (16) and better control of intracranial pressure and brain tissue partial pressure of oxygen (17), randomized clinical trials have not reliably validated these outcomes. Present meta-analyses are limited to surrogate endpoints e.g., intracranial pressure or have not noticed significant differences in death or functional result between hypertonic saline and mannitol (12–14), However, guidelines highlight that existing data are inadequate to suggest one solution over the other, and suggest that additional studies are needed in this field (4–6). So, it is still uncertain whether hypertonic saline is better than mannitol in the controlling of subjects with traumatic brain injury or not. The present meta-analysis aimed to evaluate the effect of hypertonic saline compared to mannitol for the management of elevated intracranial pressure in traumatic brain injury.

The article "Hypertonic Saline Compared to Mannitol for the Management of Elevated Intracranial Pressure in Traumatic Brain Injury: A Meta-Analysis" was retracted in 2023. Reasons: plagiarism; overlap with other authors' work; unreliable results or conclusions; concerns about the authorship.

## Materials and Methods

The present study followed the meta-analysis of studies in the epidemiology statement (18), which was performed following an established protocol.

### Study Selection

The study parameters included statistical measures of association (odds ratio [OR], mean difference [MD], frequency rate ratio, or relative risk, with 95% confidence intervals [CIs]) between the effect of hypertonic saline compared to mannitol for the management of elevated intracranial pressure in traumatic brain injury.

Inclusion was not restricted by study size or type. Publications excluded were review articles, commentaries, and studies that did not supply a degree of relationship. Figure 1 shows the whole study process.

**Figure 1:** Schematic diagram of the study procedure.

The articles were integrated into the meta-analysis when the following inclusion criteria were met:

1. The study was a randomized control trial or a retrospective study.
2. The target population includes subjects with traumatic brain injury.
3. The intervention program was the effect of hypertonic saline compared to mannitol for the management of elevated intracranial pressure in traumatic brain injury.
4. The study included comparisons between the hypertonic saline and mannitol.

The exclusion criteria for the intervention groups were:

1. Studies that did not determine the effect of hypertonic saline compared to mannitol for the management of elevated intracranial pressure in traumatic brain injury.
2. Studies that included managements of intracranial pressure after traumatic brain injury other than the effect of hypertonic saline and mannitol.
3. Studies that did not focus on the effect on comparative results.

### Identification

A protocol of search strategies was prepared according to the PICOS principle (19), and we defined it as follow: *p* (population): subjects with traumatic brain injury; I (intervention/exposure): hypertonic saline and mannitol; C (comparison): effect of hypertonic saline compared to mannitol; O (outcome): treatment failure, a favorable outcome, and mortality and changes in cerebral perfusion pressure, and intracranial pressure; and S (study design): no restriction (20). First, we conducted a systematic search of Embase, PubMed, Cochrane Library, OVID, and Google Scholar till July 2021, by using a blend of keywords and related words for the hypertonic saline, mannitol, intracranial pressure, treatment failure, cerebral perfusion pressure, traumatic brain injury, a favorable outcome, and mortality as shown in Table 1. All detected studies were gathered in an EndNote file, duplicates were removed, and the title and abstracts were revised to eliminate studies that did not show any relationship between the effects of hypertonic saline compared to mannitol for the management of elevated intracranial pressure in traumatic brain injury. The remaining studies were examined for related information.

The article "Hypertonic Saline Compared to Mannitol for the Management of Elevated Intracranial Pressure in Traumatic Brain Injury: A Meta-Analysis" was retracted in 2023. Reasons: plagiarism; overlap with other authors' work; unreliable results or conclusions; concerns about the authorship.

**Table 1:** Search strategy for each database.

**Database**	**Search strategy**
Pubmed	#1 ”hypertonic Saline“[MeSH Terms] OR ”mannitol“[All Fields] OR ”intracranial pressure“[All Fields] #2 ”traumatic brain injury“[MeSH Terms] OR ”hypertonic Saline“[All Fields] OR ”Treatment failure“[All Fields] OR ”Cerebral perfusion pressure“[All Fields] OR ”Favorable outcome“[All Fields] OR ”Mortality"[All Fields] #3 #1 AND #2
Embase	'hypertonic Saline'/exp OR 'mannitol'/exp OR 'intracranial pressure'/exp #2 'traumatic brain injury'/exp OR 'ICBG'/exp OR 'Treatment failure'/exp OR 'Cerebral perfusion pressure'/exp OR 'Favorable outcome'/exp OR 'Mortality'/exp #3 #1 AND #2
Cochrane library	#1 (hypertonic Saline):ti,ab,kw OR (mannitol):ti,ab,kw OR (intracranial pressure):ti,ab,kw (Word variations have been searched) #2 (traumatic brain injury):ti,ab,kw OR (Treatment failure):ti,ab,kw OR (Cerebral perfusion pressure):ti,ab,kw OR (Favorable outcome):ti,ab,kw OR (Mortality):ti,ab,kw (Word variations have been searched) #3 #1 AND #2

### Screening

Data were abridged onto a standardized form on the following basis; study-related and subject-related characteristics as follows: last name of the primary author, period of study, year of publication, country, region of the studies, and study design; population type, the total number of subjects, demographic data and clinical and treatment characteristics; categories, qualitative and quantitative method of evaluation, information source, and outcome evaluation; and statistical analysis (21). If a study qualified for inclusion based upon the aforementioned principles, data were extracted independently by two authors. In case of disagreement, the corresponding author provided a final opinion. When the data from a particular study differed based on the assessment of the relationship between the effects of hypertonic saline compared to mannitol for the management of elevated intracranial pressure in traumatic brain injury, we extracted the data separately. There is a risk of bias in these studies; therefore, individual studies were evaluated using two authors who independently assessed the methodological quality of the selected studies. The “risk of bias tool“ from the RoB 2: A revised Cochrane risk-of-bias tool for randomized trials was utilized to evaluate methodological quality (22). In terms of the evaluation criteria, each study was evaluated and allocated to one of the next three risks of bias-low: if all quality criteria were met, the study was considered to have a low risk of bias; unclear: if one or more of the quality criteria were partially met or unclear, the study was considered to have a moderate risk of bias; or high: if one or more of the criteria were not met, or not included, the study was considered to have a high risk of bias. Any discrepancies were addressed by a reassessment of the original article.

The article "Hypertonic Saline Compared to Mannitol for the Management of Elevated Intracranial Pressure in Traumatic Brain Injury: A Meta-Analysis" was retracted in 2023. Reasons: plagiarism; overlap with other authors' work; unreliable results or conclusions; concerns about the authorship.

### Eligibility

The main result concentrated on the effect of hypertonic saline compared to mannitol for the management of elevated intracranial pressure in traumatic brain injury. An assessment of these aforementioned effects in subjects with traumatic brain injury was summarized.

### Inclusion

Sensitivity analyses were limited to studies reporting the relationship between the effects of hypertonic saline compared to mannitol for the management of elevated intracranial pressure in traumatic brain injury. For subcategory and sensitivity analysis, we compared the hypertonic saline and mannitol.

### Statistical Analysis

We calculate the odds ratio (OR), mean difference (MD), and 95% confidence interval (CI) using the dichotomous or continuous method with a random or fixed-effect model. We calculated the I^2^ index and the I^2^ index was ranging from 0 to 100%. When the I^2^ index was ~0, 25, 50, and 75% that specifies no, low, moderate, and high heterogeneity, respectively (19). If the I^2^ was >50%, we used the random-effect; if it was <50%, we used the fixed-effect. We stratified the original assessment as per result categories as described previously to complete the subgroup analysis. Differences among the subcategories were considered statistically significant at a *p*-value < 0.05. Publication bias was assessed quantitatively using the Egger regression test (publication bias is present if *p* ≥ 0.05), and qualitatively, by visual inspection of funnel plots of the logarithm of odds ratios vs. their standard errors (21). All the *p*-values were calculated *via* two-tailed tests. Reviewer manager version 5.3 (The Nordic Cochrane Centre, The Cochrane Collaboration, Copenhagen, Denmark) was used to do all calculations and graphs.

## Results

A total of 743 unique studies were identified, of which 17 studies (between 2003 and 2021) fulfilled the inclusion criteria and were included in this meta-analysis (23–39). The 17 studies included 1,392 subjects with traumatic brain injury at the start of the study; 708 of them were administered hypertonic saline and 684 were given mannitol. All studies evaluated the effect of hypertonic saline compared to mannitol for the management of elevated intracranial pressure in traumatic brain injury.

The article "Hypertonic Saline Compared to Mannitol for the Management of Elevated Intracranial Pressure in Traumatic Brain Injury: A Meta-Analysis" was retracted in 2023. Reasons: plagiarism; overlap with other authors' work; unreliable results or conclusions; concerns about the authorship.

The study size ranged from 20 to 457 subjects with traumatic brain injury at the start of the study. The details of the 17 studies are shown in Table 2. Five studies reported data stratified to the changes in treatment failure, 14 studies reported data stratified to the changes in intracranial pressure, 7 studies reported data stratified to the changes in cerebral perfusion pressure, 6 studies reported data stratified to the favorable outcome, and 7 studies reported data stratified to the mortality in subjects with traumatic brain injury.

**Table 2:** Characteristics of the selected studies for the meta-analysis.

**Study**	**Country**	**Total**	**Hypertonic saline**	**Mannitol**
Vialet et al. (23)	France	20	10	10
Harutjunyan et al. (24)	Germany	32	17	15
Mao et al. (25)	China	56	28	28
Francony et al. (26)	USA	20	10	10
Oddo et al. (27)	USA	22	11	11
Kerwin et al. (28)	USA	22	11	11
Ichai et al. (29)	France	33	17	16
Cottenceau et al. (30)	France	47	22	25
Sakellaridis et al. (31)	Greece	64	32	32
Hendoui et al. (32)	Iran	33	23	10
Huang et al. (33)	India	238	119	119
Jagannatha et al. (34)	India	38	18	20
Du et al. (35)	China	132	65	67
Qin et al. (36)	China	48	24	24
Patil et al. (37)	India	80	40	40
Huang et al. (38)	China	457	236	221
Mangat et al. (39)	USA	50	25	25
	Total	1,392	708	684

Hypertonic saline had significantly lower treatment failure (OR, 0.38; 95% CI, 0.15–0.98, *p* = 0.04) with moderate heterogeneity (I^2^ = 50%), lower intracranial pressure 30–60 mins after infusion termination (MD, −1.12; 95% CI, −2.11 to −0.12, *p* = 0.03) with high heterogeneity (I^2^ = 85%), and higher cerebral perfusion pressure 30–60 mins after infusion termination (MD, 5.25; 95% CI, 3.59–6.91, *p* < 0.001) with high heterogeneity (I^2^ = 94%) compared to mannitol in subjects with traumatic brain injury as shown in Figures 2–4.

**Figure 2:** Forest plot of the treatment failure of hypertonic saline compared to mannitol when used for the management of elevated intracranial pressure in traumatic brain injury.

**Figure 3:** Forest plot of the effect of hypertonic saline compared to mannitol on intracranial pressure 30–60 mins after infusion termination when used for the management of elevated intracranial pressure in traumatic brain injury.

**Figure 4:** Forest plot of the effect of hypertonic saline compared to mannitol on cerebral perfusion pressure 30–60 mins after infusion termination when used for the management of elevated intracranial pressure in traumatic brain injury.

The article "Hypertonic Saline Compared to Mannitol for the Management of Elevated Intracranial Pressure in Traumatic Brain Injury: A Meta-Analysis" was retracted in 2023. Reasons: plagiarism; overlap with other authors' work; unreliable results or conclusions; concerns about the authorship.

However, hypertonic saline had no significant effect on favorable outcome (OR, 1.61; 95% CI, 1.01–2.58, *p* = 0.05) with low heterogeneity (I^2^ = 37%), mortality (OR, 0.59; 95% CI, 0.34–1.02, *p* = 0.06) with no heterogeneity (I^2^ = 0%), intracranial pressure 90–120 mins after infusion termination (MD, −0.90; 95% CI, −3.21–1.41, *p* = 0.45) with high heterogeneity (I^2^ = 95%), cerebral perfusion pressure 90–120 mins after infusion termination (MD, 4.28; 95% CI, −0.16–8.72, *p* = 0.06) with high heterogeneity (I^2^ = 97%), and duration of elevated intracranial pressure per day (MD, 2.20; 95% CI, −5.44–1.05, *p* = 0.18) with high heterogeneity (I^2^ = 97%) compared to mannitol in subjects with traumatic brain injury as shown in Figures 5–9.

**Figure 5:** Forest plot of the favorable outcome of hypertonic saline compared to mannitol when used for the management of elevated intracranial pressure in traumatic brain injury.

**Figure 6:** Forest plot of the mortality of hypertonic saline compared to mannitol when used for the management of elevated intracranial pressure in traumatic brain injury.

**Figure 7:** Forest plot of the effect of hypertonic saline compared to mannitol on intracranial pressure decrease 90–120 mins after infusion termination when used for the management of elevated intracranial pressure in traumatic brain injury.

**Figure 8:** Forest plot of the effect of hypertonic saline compared to mannitol on cerebral perfusion pressure 90–120 mins after infusion termination when used for the management of elevated intracranial pressure in traumatic brain injury.

**Figure 9:** Forest plot of the duration of elevated intracranial pressure per day of hypertonic saline compared to mannitol when used for the management of elevated intracranial pressure in traumatic brain injury.

Selected studies stratified analysis that did and did not adjust for age, gender, and ethnicity were not performed, since no studies reported or adjusted for these factors.

Based on the visual inspection of the funnel plot as well as on quantitative measurement using the Egger regression test, there was no evidence of publication bias (*p* = 0.89). However, most of the included studies were assessed to be of low methodological quality due to their small sample size. All studies did not have selective reporting bias, and no articles had incomplete outcome data and selective reporting.

## Discussion

This meta-analysis study based on the 17 studies included 1,392 subjects with traumatic brain injury at the start of the study; 708 of them were administered hypertonic saline and 684 were given mannitol (23–39). Hypertonic saline had significantly lower treatment failure, lower intracranial pressure 30–60 mins after infusion termination, and higher cerebral perfusion pressure 30–60 mins after infusion termination compared to mannitol in subjects with traumatic brain injury. However, hypertonic saline had no significant effect on the favorable outcome, mortality, intracranial pressure 90–120 mins after infusion termination, cerebral perfusion pressure 90–120 mins after infusion termination, and duration of elevated intracranial pressure per day compared to mannitol in subjects with traumatic brain injury (23–39). Hence, the most relevant question, namely whether hypertonic saline might be superior to mannitol in improving the outcome after the head injury, remains unanswered since most of the outcomes showed no significant difference. This could be due to the high biases potentially contributed by some of the included studies e.g., the study by Vialet et al. (23) that could affect the results very much. Though, the analysis of results should be done with carefulness due to the low number of studies for some parameters studied e.g., for a favorable outcome, mortality, and cerebral perfusion pressure 90–120 mins after infusion termination and the low sample size in most of the included studies (14 studies ≤ 100 subjects) in the meta-analysis; recommending the requirement for more studies to confirm these findings or probably to significantly affect the confidence in the effect assessment especially for the favorable outcome, mortality, and cerebral perfusion pressure with their very low *p*-value (*p* = 0.05, 0.06, and 0.06).

The article "Hypertonic Saline Compared to Mannitol for the Management of Elevated Intracranial Pressure in Traumatic Brain Injury: A Meta-Analysis" was retracted in 2023. Reasons: plagiarism; overlap with other authors' work; unreliable results or conclusions; concerns about the authorship.

Intracranial hypertension produced by traumatic brain injury could result in numerous dangers, e.g., cerebral ischemia, Cushing reaction, brain shift, and neurogenic pulmonary edema (40). Intracranial hypertension is defined in the past as intracranial pressure>20 mmHg, a value that is an accepted standard for initiating clinical interference. Intracranial pressure is a major predictor of neurologic worsening in subjects with traumatic brain injury (41). It has also been shown that if cerebral perfusion pressure is extremely low (<50 mm Hg), intracranial pressure becomes a predictor of the poor result, and keeping intracranial pressure in the range of 18 to 23 mmHg confirms that cerebral perfusion pressure remains stable for a longer time (42). Mannitol has been used to decrease raised intracranial pressure for many years. Recently it was suggested by guidelines that mannitol is more effective in decreasing intracranial pressure in subjects with traumatic brain injury compared with barbiturates (5). However, mannitol has its side effects e.g., pulmonary edema, acute renal failure, rebound cerebral edema, aggravation, and arterial hypotension causing a reduction in cerebral perfusion pressure by its diuretic effect (14), the best therapeutic agent to manage intracranial pressure should decrease intracranial pressure though keeping cerebral perfusion. Hypertonic saline adverse effects are seldom reported e.g., continuous infusing hypertonic saline sustains the serum sodium concentration to 170 mmol/L and was related to neutropenia, acute renal failure, thrombocytopenia, acute respiratory distress syndrome, and anemia (43). Hypertonic saline significantly raises serum sodium and osmolality. Excessive increases in sodium levels and osmolarity cause volume overload with pulmonary edema and heart failure or could initiate coagulopathy, and hyperchloremic metabolic acidosis (44, 45). Thus, the hypertonic solutions used in subjects with diminished cardiac function should be done with caution and under close cardiac monitoring. Similar to our results intravenous use of hypertonic saline improved cerebral perfusion and caused a shift of the oxygen dissociation curve, so improving oxygen supply, and brain compliance, and reducing cerebral edema, and intracranial pressure (46). However, proofs on the hypertonic saline use in severe traumatic brain injury are imperfect in showing its advantage in decreasing intracranial pressure and mortality (42).

There is proof that episodes of cerebral perfusion pressure <60 mmHg or intracranial pressure >20 mmHg are related to a poorer result, and that cerebral perfusion pressure ≥70 mmHg by treatment is an accepted management goal (5). The change in the level of significance when using hypertonic saline compared to mannitol in lowering intracranial pressure, and improving cerebral perfusion pressure 30–60 mins after infusion termination to insignificance 90–120 mins after infusion termination is worth further evaluation. It was shown before that the intracranial pressure returned to pretreatment levels after a median time of 90 mins (47). However, when mannitol was administered at a slower rate (20–30 mins), no intracranial pressure rebound was observed in 2 h after infusion. This recommends that the duration of the mannitol effect might be affected by the infusion rate; the quicker the infusion, the faster the termination of the effect by the rapid renal removal or diffusion of mannitol into the brain tissue. Also, the strength, route of administration of hypertonic saline or mannitol timing, and frequency require to be evaluated in a large multicenter study.

The article "Hypertonic Saline Compared to Mannitol for the Management of Elevated Intracranial Pressure in Traumatic Brain Injury: A Meta-Analysis" was retracted in 2023. Reasons: plagiarism; overlap with other authors' work; unreliable results or conclusions; concerns about the authorship.

This meta-analysis showed the relationship between the effects of hypertonic saline compared to mannitol for the management of elevated intracranial pressure in traumatic brain injury. However, further studies are needed to validate these potential associations. Also, further studies are needed to deliver a clinically meaningful difference in the results. This was also suggested in another meta-analysis which showed a similar effect of hypertonic saline and mannitol for the management of elevated intracranial pressure in subjects with traumatic brain injury (12–14). Well-designed studies are also needed to assess these factors including the combination of different ages, gender, and ethnicity; since our meta-analysis study could not answer whether these factors are associated with the results (48). In summary, Hypertonic saline had significantly lower treatment failure, lower intracranial pressure 30–60 mins after infusion termination, and higher cerebral perfusion pressure 30–60 mins after infusion termination compared to mannitol in subjects with traumatic brain injury. However, hypertonic saline had no significant effect on the favorable outcome, mortality, intracranial pressure 90–120 mins after infusion termination, cerebral perfusion pressure 90–120 mins after infusion termination, and duration of elevated intracranial pressure per day compared to mannitol in subjects with traumatic brain injury. Further studies are required to validate these findings.

### Limitations

There may be a selection bias in this study since so many of the studies found were excluded from the meta-analysis. However, the studies excluded did not satisfy the inclusion criteria of our meta-analysis. Moreover, we could not determine if the results were associated with age, gender, and ethnicity or not. The study designed to assess the relationship between the effects of hypertonic saline compared to mannitol was based on data from previous studies, which might cause bias due to incomplete details. The meta-analysis was based on 17 studies with a low number of studies for some parameters e.g., for a favorable outcome, mortality, intracranial pressure 90–120 mins after infusion termination, and cerebral perfusion pressure 90–120 mins after infusion termination and the low sample size in most of the selected studies (14 studies ≤ 100 subjects). Factors including the age, gender, compliance, ethnicity, and nutritional status of patients were also possible bias-inducing factors. Some unpublished studies and missing data may cause a bias in the pooled effect. Patients were using different management schedules, dosages, and health care systems.

The article "Hypertonic Saline Compared to Mannitol for the Management of Elevated Intracranial Pressure in Traumatic Brain Injury: A Meta-Analysis" was retracted in 2023. Reasons: plagiarism; overlap with other authors' work; unreliable results or conclusions; concerns about the authorship.

## Conclusions

Hypertonic saline had significantly lower treatment failure, lower intracranial pressure 30–60 mins after infusion termination, and higher cerebral perfusion pressure 30–60 mins after infusion termination compared to mannitol in subjects with traumatic brain injury. However, hypertonic saline had no significant effect on the favorable outcome, mortality, intracranial pressure 90–120 mins after infusion termination, cerebral perfusion pressure 90–120 mins after infusion termination, and duration of elevated intracranial pressure per day compared to mannitol in subjects with traumatic brain injury. However, the analysis of results should be done with carefulness due to the low number of studies for some parameters and the low sample size in most of the included studies in the meta-analysis; recommending the requirement for more studies to confirm these findings or probably to significantly affect the confidence in the effect assessment.

## Data Availability Statement

The original contributions presented in the study are included in the article/supplementary material, further inquiries can be directed to the corresponding author/s.

## Author Contributions

JZ: conception and design. CH, FY, and SG: collection and assembly of data. CH, FY, SG, and JZ: administrative support, provision of study materials or subjects, data analysis and interpretation, manuscript writing, and final approval of manuscript. All authors have read and approved the manuscript.

## Funding

This research was supported by Medical Youth Support Project of PLA General Hospital: QNF19028.

## Conflict of Interest

The authors declare that the research was conducted in the absence of any commercial or financial relationships that could be construed as a potential conflict of interest.

## Publisher's Note

All claims expressed in this article are solely those of the authors and do not necessarily represent those of their affiliated organizations, or those of the publisher, the editors and the reviewers. Any product that may be evaluated in this article, or claim that may be made by its manufacturer, is not guaranteed or endorsed by the publisher.
